# Mining of Potential Biomarkers and Pathway in Valvular Atrial Fibrillation (VAF) via Systematic Screening of Gene Coexpression Network

**DOI:** 10.1155/2022/3645402

**Published:** 2022-10-03

**Authors:** Fan Zou, Tiantian Chen, Xiuying Xiang, Chengjiang Peng, Shuai Huang, Shaohong Ma

**Affiliations:** ^1^Department of Cardiovascular Surgery, The Third Affiliated Hospital of Sun Yat-sen University, No. 600, Tianhe Road, Tianhe District, Guangzhou City, Guangdong Province, China; ^2^Department of Hematopathology, The First Affiliated Hospital of Jinan University, Tianhe District, Guangzhou City, Guangdong Province, China

## Abstract

**Purpose:**

We apply the bioinformatics method to excavate the potential genes and therapeutic targets associated with valvular atrial fibrillation (VAF).

**Methods:**

The downloaded gene expression files from the gene expression omnibus (GEO) included patients with primary severe mitral regurgitation complicated with sinus or atrial fibrillation rhythm. Subsequently, the differential gene expression in left and right atrium was analyzed by R software. Additionally, weighted correlation network analysis (WGCNA), principal component analysis (PCA), and linear model for microarray data (LIMMA) algorithm were used to determine hub genes. Then, Metascape database, DAVID database, and STRING database were used to annotate and visualize the gene ontology (GO) analysis, KEGG pathway enrichment analysis, and PPI network analysis of differentially expressed genes (DEGs). Finally, the TFs and miRNAs were predicted by using online tools, such as PASTAA and miRDB.

**Results:**

20,484 differentially expressed genes related to atrial fibrillation were obtained through the analysis of left and right atrial tissue samples of GSE115574 gene chip, and 1,009 were with statistical significance, including 45 upregulated genes and 964 downregulated genes. And the hub genes implicated in AF of NPC2, ODC1, SNAP29, LAPTM5, ST8SIA5, and FCGR3B were screened. Finally, the main regulators of targeted candidate biomarkers and microRNAs, EIF5A2, HIF1A, ZIC2, ELF1, and STAT2, were found in this study.

**Conclusion:**

These hub genes, NPC2, ODC1, SNAP29, LAPTM5, ST8SIA5, and FCGR3B, are important for the development of VAF, and their enrichment pathways and TFs elucidate the involved molecular mechanisms and assist in the validation of drug targets.

## 1. Background

Atrial fibrillation (AF) is the most common sustained arrhythmia, and actual epidemiological data are often underestimated. According to research, in China, the prevalence and incidence of atrial fibrillation show increasing epidemiological characteristics with age, and the total prevalence of the population can reach 0.77%, and those over 80 years old can reach over 10 years old [1]. With the development of my country's economy and the aging of the population, the number of patients with atrial fibrillation has increased rapidly, and the number of patients with atrial fibrillation is expected to increase exponentially in the next 10 years [2]. Embolism and heart failure are common complications of atrial fibrillation, and the mortality rate is more than twice that of the general population [3]. Due to the numerous pathogenic factors of atrial fibrillation, it is difficult to prevent and treat clinically, which is still one of the problems in cardiovascular.

Valve disease is one of the common causes of atrial fibrillation in cardiovascular surgery, including macrovascular disease, congenital heart disease, and coronary artery disease [4]. Valvular atrial fibrillation was first proposed in the 2012 ESC updated guidelines, in which atrial fibrillation is divided into “valvular atrial fibrillation (VAF)” and “nonvalvular atrial fibrillation (NVAF)”, VAF is defined as valvular heart disease atrial fibrillation and atrial fibrillation, fibrillation after valve replacement [5]. Common complications of atrial fibrillation include heart failure and embolism. The study found that the incidence of heart failure caused by atrial fibrillation is 3.4 times that of normal people, while the incidence of embolism caused by atrial fibrillation is about 5% per year, which is 7 times that of normal people [6]. Cerebral embolism is the most common and most dangerous complication of atrial fibrillation. Studies have shown that the incidence of stroke caused by atrial fibrillation is 20% per year. The stroke caused by NVAF is 7 times that of normal people, while the stroke caused by VAF is up to 17 times that of normal people [7]. According to the survey, the incidence of valvular atrial fibrillation is as high as 70%, and the mortality and disability rate caused by heart failure and cerebral embolism are higher in cardiac surgery complicated with atrial fibrillation. Valvular atrial fibrillation seriously affects the hospitalization time and survival time of patients, seriously reduces the quality of life of patients, and also brings serious economic burden to family members. However, current treatments have not achieved satisfactory results [8]. In view of its high incidence and serious impact on human health and safety, exploring the diagnosis and treatment of valvular atrial fibrillation is one of the research hotspots in the cardiovascular field in recent years.

At present, the treatment of atrial fibrillation is generally divided into drug therapy and nondrug therapy. Drug therapy mainly includes ventricular rate control, anticoagulation therapy to prevent thromboembolism, and antiarrhythmic therapy to restore and maintain sinus rhythm. Long-term drug therapy has a high recurrence rate, which leads to new-onset arrhythmias, and also brings many disadvantages to patients, such as poor tolerance, bleeding risk caused by anticoagulant drugs, and poor efficacy. In interventional therapy, radiofrequency ablation has become one of the most important methods for the treatment of valvular atrial fibrillation. However, there are still some deficiencies in radiofrequency ablation for atrial fibrillation, the recurrence rate is still high, up to 40%, and with the extension of follow-up time, the recurrence rate is still on the rise [9–11]. Therefore, the key to solving the problem lies in elucidating the molecular mechanism of the occurrence and maintenance of valvular atrial fibrillation. Whether there are key regulatory factors in the process has not been reported.

However, the genetic variants currently defined combine to explain only a small fraction of the incidence of atrial fibrillation. On the one hand, many studies have focused on serum and animal experiments to explore the relationship between atrial fibrillation and mechanisms or biomarkers, but there are fewer reports on atrial tissue directly affecting atrial fibrillation, especially in patients with valvular atrial fibrillation. On the other hand, these results suggest that genetic variants isolated from individual samples cannot be broadly applied to the general population. Hub genes identified from differential expression analysis may lose statistical power in protein-protein interaction networks due to mutual functional regulation. Due to the high standard of genetic selection, some key genes may have been lost. Based on the above notes, we will use multiple algorithms, including LIMMA, WGCN, PCA, and gene functional analysis of microarray data, to obtain key genes and gene regulatory networks for valvular atrial fibrillation. These will help us better understand the molecular mechanism of atrial fibrillation and the interaction of the complex gene environment and provide a theoretical basis for the diagnosis and treatment of atrial fibrillation.

## 2. Materials and Methods

### 2.1. Materials

We downloaded these data from the Public Resource Database GEO (http://www.ncbi.nlm.nih.gov/geo/) and generated expression profiling arrays using Affymetrix Human Genome U133 Plus 2 GPL570 (HG-U133_Plus_2). The retrieval involved the following process: (1) collecting datasets searched with the keywords “atrial fibrillation” and “valvular disease”. (2) Select “Homo sapiens” as the specimen source and “Expression profiling by high throughput sequencing” as the study type. (3) The gene chip data is selected as “Affymetrix Human Genome” on the test platform. The GSE115574 dataset was published on September 4, 2019, from surgically resected left and right atrial tissue from 30 patients with severe chronic mitral regurgitation, including 15 with preoperative atrial fibrillation and 15 with preoperative sinus. In this study, patients with persistent atrial fibrillation lasted more than 6 months. Patients with sinus rhythm had no clinical evidence of atrial fibrillation and no history of any antiarrhythmic drugs.

### 2.2. Data Processing

Using the “ComBat” function of the SVA package, the study is aimed at eliminating bias from the high-throughput data from different microarrays. The aim of bioinformatics is to analyze all of the raw data from microarrays, including background correction, quantile normalization, and probe summarization values [12]. The study also used some advanced algorithms, such as robust multiarray average for background-adjusted, normalized, and log-transformed probe expression values; the *t*-test in the “LIMMA” package to identify differentially expressed genes (DEGs); and the Benjamini–Hochberg method that aims at adjusting *P* values [13]. DEGs are gene expression values with ∣ log2FC | >1 and *P* value <0.05. The aim of selecting coannotated genes (a total of 20,484 genes) in GPL570 platform was to illuminate further coexpression network analysis.

### 2.3. Weighted Gene Coexpression Network (WGCN) Construction and Module Detection

The coexpression network analysis has functions which integrate other informations and avoid information missing. Another system-level insight is better than other approaches, so as to give WGCNA an edge. Therefore, a system-level analysis based on WGCNA is used in the study. The WGCN was constructed using the WGCN package in RStudio. All analyses were conducted using RStudio [14].

The functional enrichment of differentially expressed genes related to atrial fibrillation was analyzed by online public database, Metascape database (http://metascape.org/gp/index.html), and database for annotation, visualization, and integrated discovery bioinformatics resources database (DAVID, http://david.abcc.ncifcrf.gov/). The analysis involved the following processes: (1) the purpose of this project is to obtain gene annotations, visualize bioinformatics resources, and integrate them, DAVID database was used to carry out gene ontology (GO) analysis on differentially expressed genes, and GO entries with *P* value less than 0.05 were considered to be significantly enriched [15]. (2) Downloaded from Metascape, the Kyoto Encyclopedia of Genes and Genomes (KEGG) pathway, and adjusted *P* value <0.05 and enrichment score > 1.0 was considered to indicate a statistically significant difference [16].

### 2.4. Construction of Protein-Protein Interaction (PPI) Network and Screening of Key Genes

Protein-protein interaction network is a complex interaction and communication network between two or more proteins. The network can take place in many biological processes, including gene expression, molecular transport, signal transduction, and catalytic metabolic reactions. It can also be used to predict the interaction between related genes and their proteins and has certain significance for studying the molecular mechanism and drug targets in the occurrence and development of diseases. Therefore, we utilize the STRING database (V10.5; http://string-db.org) and Cytoscape software (V3.5.1; http://cytoscape.org/) to construct PPI network of differentially expressed genes enriched in key KEGG pathway, such as biological metabolic processes, autophagy, ion conversion, and immune inflammatory processes and to visualize and annotate. The cut-off criteria were set to: *P* < 0.05 and enrichment score > 1.0, that is, the elimination of no correlation or weak action of the protein [17]. We obtain the key modules and core genes in PPI network using the MCODE plugin of Cytoscape software.

### 2.5. Prediction of Transcription Factors and microRNAs of Key Genes

The transcription factors of key genes are predicted by using the iRegulon plugin of the Cytoscape software, and the parameters are set as follows: the minimum value of gene homology is 0.05; maximum FDR for motif similarity is 0.001; and the normalized enrichment score (NES) is greater than 5. Finally, using online tools from miRDB (http://mirdb.org/) was applied to predict interactions between miRNAs and co-DEGs involved in AF. Therefore, the regulatory factors with high NSE values and microRNAs were used as regulatory networks to participate in the development of atrial fibrillation.

## 3. Results

### 3.1. Identification of Differentially Expressed Genes (DEGs)

The AF and SR patients without additional treatment from GSE115574 (GPL570) datasets were used in all the samples for further analysis, including 15 cases of preoperative atrial fibrillation and 15 cases of preoperative sinus. We identified 54,675 probes corresponding to 20,484 genes in GSE115574 datasets and GPL570 platform. There were 1,009 DEGs with statistical significance, including 45 upregulated genes and 964 downregulated genes. The first five genes of up- and downregulated genes are shown in Table 1. The heat map and the volcano plot for the DEGs are illustrated in Figure 1.

### 3.2. Construct Coexpression Network and Gene Module

We obtained 6 clusters (MElightcyan, MEgrey, MEmagenta, MEred, MEturquoise, and MEyellow; Figure 2(a)) in the 59 samples with 1009 gene variables after sample cluster analysis and samples that did not get lost in the analyses. The WGCN analysis involved the following processes: (1) when the standard parameter was set to 10 (power valve), the scale independence rose to 0.8 and the mean relation was higher in Figure 2(b). (2) We obtained the two key models, MElightcyan: VAF Pearson valve = 0.97, *P* = 1*e* − 38; SR Pearson valve = −0.97, *P* = 1*e* − 38 and MEturquoise: VAF Pearson valve = 0.86, *P* = 4*e* − 18; SR Pearson valve = −0.86, *P* = 4*e* − 18 (Figure 2(c)). (3) The heat map suggested no significant difference in module genes. The interaction analysis of coexpression modules showed a significant independence (Figure 2(d)). (4) We found the three clusters in different modules of the connectivity of eigen-genes, and the study illuminates obvious connectivity among the eigen-genes of different modules within the same cluster showed, whereas there was no difference among different clusters' modules in Figure 2(d). (5) Differentially expressed genes in the MElightcyan and MEturquoise modules are shown in Table 2. On other hand, as to VAF, we also found the significant difference of the MEgreen and MEbrown module genes in response to AF and SR in two-dimensional PCA results (Figure 2(e)). Figures 2(f) and 2(g) show the gene significance (GS) analysis results about a significant difference between the genes and the characteristic of AF, *P* values are far less than 0.05.

### 3.3. Functional GO Terms and Pathway Enrichment Analyses

Further functional enrichment analysis was carried out on DEGs of the MElightcyan and MEturquoise key modules, including gene ontology (GO) analysis and KEGG pathway enrichment analysis. Regarding GO terms enrichment, the MElightcyan module was mainly enriched in GO biological process (BP): cell protein modification process, intracellular signal transduction process, proteasome-mediated ubiquitin-dependent protein degradation process, negative regulation of classical Wnt signaling pathway, stimulating c-type lectin receptor signaling pathway, and other common processes such as enrichment. Cellular components: cytoplasm, extracellular matrix, cell membrane, Golgi body, endoplasmic reticulum, mitochondria, etc. Molecular function: protein binding, ATP energy binding, transmembrane transport, same protein binding point, ubiquitin protein transferase activity, protein activation, etc. These results are shown in Figure 3(a). Genes in the MEturquoise module were predominantly enriched in BP: vesicle secretion, cell localization, membrane tissue generation, membrane protein localization, etc. In terms of cellular components, genes are mainly enriched in membrane components, including plasma membrane and extracellular membrane. In terms of MF, it is mainly concentrated in the activity of energy receptor and amino acid transmembrane transporter. These results are illustrated in Figure 3(b).

KEGG pathway analysis data appeared in Figure 4 is downloaded to the Metascape database. The results suggested that the MElightcyan module genes were significantly enriched in the interaction of vesicular transport, classical mTOR signaling pathway, FOXO signaling pathway, biosynthesis, and metabolism. MEturquoise module DEGs are enriched in natural killer cell-mediated cytotoxicity, cytoskeleton synthesis, and inflammatory response pathways.

### 3.4. Construction of Protein-Protein Interaction (PPI) Network and Screening of DEGs

Additionally, Table 3 illustrates a part of the visible pathway that is tightly correlated with atrial structural remodeling and electrical remodeling from the KEGG pathway network. After submitting the genes enriched in cancer-correlated pathways to the STRING database, PPI network were obtained for the MElightcyan and MEturquoise modules, respectively, with a confidence threshold greater than 0.4 in Figure 5(a). We subsequently conducted a module analysis. When a “score > 3” was defined as the cut-off criterion in MCODE, 5 clusters of modules (Module 1, Module 2, Module 3, Module 4, and Module 5) were identified from the PPI network visualized by STRING in the MElightcyan modules (Figures 5(b)–5(f)), and Figure 5(g) shows the functional modules of the MEturquoise modules. Furthermore, the MCODE analysis showed the 6 seed genes of each cluster, these were ST8SIA5, ODC1, LAPTM5, NPC2, SNAP29, and FCGR3B. Thus, they are likely to be novel therapeutic target genes or biomarkers.

### 3.5. Identification of Hub Gene Involving in VAF

What's more, the gene expression levels in clinical traits and left or right atrial tissues were compared based on GEO database. Consequently, the gene differential expression level with regrading to hub genes was constructed. We also found a statistical difference in the gene expression levels of these genes between VAF and SR, while no statistical difference between right and left atrial tissues in Figure 6. Subsequently, expression levels of the six hub genes show a significant difference in expression level between VAF and SR, respectively.  Figure 7 appeared all the *P* < 0.05.

### 3.6. Investigating Transcription Factors (TFs) and microRNAs of Hub Genes

To extend our findings, we predicted the TFs and found that EIF5A2, HIF1A, ZIC2, ELF1, and STAT2 as the master regulators of the hub genes are involved in VAF. The results are illustrated in Table 4 and Figure 8. Finally, prediction analysis using miRDB and TargetScan bioinformatic tools identified the selected miRNAs targeting each hub co-DEG involved in AF and these data appear. These data enable us to understand how predicted miRNAs are related to AF progress and maintain.

## 4. Discussion

Currently, the pathogenesis of atrial fibrillation is still unclear, but atrial electrical remodeling and atrial structural remodeling are considered as important pathological mechanisms for the occurrence and maintenance of atrial fibrillation. Due to the reversibility of electrical remodeling and the irreversibility of structural remodeling, it is of vital significance to study atrial structural remodeling for the occurrence, development, diagnosis, and treatment of AF [18, 19]. Atrial fibrosis is not only the characteristic manifestation of atrial structural remodeling but also the primary prerequisite for the occurrence and maintenance of atrial fibrillation. Therefore, the molecular mechanism of atrial fibrosis may be a potential target for the treatment of AF [20]. The present study suggests that these mechanisms may be involved in the process of atrial fibrosis leading to atrial fibrillation, including renin-angiotensin-aldosterone system (RAAS), transforming growth factor-*β*1 (TGF-*β*1), oxidative stress and inflammation, calcium overload, MMPs, and microRNA.

Some research teams have found that RAAS system plays an important role in atrial electrical remodeling and structural remodeling, participating in various arrhythmia and atrial fibrosis processes [21]. Under physiological conditions, the core factor of RAAS is Ang-II, which physiologically can contract blood vessels, raise hypertension, and increase cardiac afterload, thus leading to cardiac structural remodeling. Xiao et al. found that Ang-II can cause obvious atrial enlargement and atrial fibrosis in mice and finally cause AF [22]. Savelieva et al. and Girmatsion et al. also found that in animal experiments, RAAS inhibitor inhibition can not only inhibit atrial remodeling and fibrosis but also delay the occurrence of atrial fibrillation; in clinical trials, angiotensin inhibitor can also reduce the incidence of new AF [23, 52]. Some studies have further found that atrial fibrosis can be caused by increasing Ang-II expression via stimulating angiotensin type 1 receptor (AT1R) and TGF-*β*1, thus leading to atrial fibrillation [24]. Transforming growth factor-*β*1 is secreted by cardiac fibroblasts and then differentiated into active fibroblasts. Atrial fibrosis is closely related to active fibroblasts. Therefore, a large number of studies show that transforming growth factor-*β*1 plays an important role in the occurrence and development of AF. Studies have found that the transforming growth factor-*β*1 is secreted not only by fibroblasts but also by macrophages, and the transforming growth factor-*β*1 can increase cell adhesion factor, which can lead to myocardial fibrosis and cardiac structural remodeling [25]. Verheule et al. found in mouse model that the stimulation of TGF-*β*1 can cause atrial fibrillation [26]. Studies have further found that the TGF-*β*1 can participate in Smad signaling pathway by regulating the expression of TGF-*β*1 activated kinase and TGF-*β*1-fibroblast protein kinase C-alpha (PKC-alpha) pathway by regulating the expression of alpha-SMA to affect atrial fibrosis and structural remodeling and lead to AF [27, 28]. Oxidative stress and inflammatory response pathway can also lead to atrial fibrosis, which in turn leads to atrial fibrillation. Some people believe that reactive oxygen species lead to atrial fibrosis and atrial fibrillation by stimulating the expression of MMPs to make fibroblast proliferation [29]. Some also believe that reactive oxygen species cause atrial fibrosis by affecting energy proteins such as nicotinamide adenine dinucleotide phosphate (NADPH) oxidase [30]. And Colman et al. found that there were a large number of inflammatory cell infiltration in fibrotic and necrotic cardiomyocytes in the atrial tissue of patients with persistent atrial fibrillation, such as Ang-II, tumor necrosis factor-*α* (TNF-*α*), interleukin- (proinflammatory cytokines and hormone release IL-) 6 and IL-8 [31].What's more, it is found that the incidence of atrial fibrillation increases with the increase of C-reactive protein, indicating that C-reactive protein can be used as an independent risk factor for atrial fibrillation [32]. On the one hand, ion channels can affect cardiac contraction by affecting cardiac electrical activity; on the other hand, it can also cause atrial fibrosis and maintain arrhythmias by delayed triggering of myocardial depolarization through a variety of pathways, such as the expression of neutral protease calpain, the activation of RyR receptors, and the opening and closing of transient receptor potential channels [33, 34]. Regarding matrix metalloproteinases (MMP), it is a family of zinc-dependent proteolytic enzymes that affect extracellular matrix, including gelatinase, collagenase, and matrix enzyme, while extracellular matrix plays an important role in the treatment of atrial fibrosis. Studies have found that tissue inhibitors of metalloproteinases (TIMPs) can affect the expression level of metalloproteinases. Now it is mainly found that metalloproteinase-2 and metalloproteinase-9 are closely related to atrial fibrosis and atrial fibrillation [35].

To this end, the research team used the GO and KEGG pathways of atrial fibrosis and atrial remodeling related to atrial fibrillation as the modules for screening candidate genes, such as ion channels, protein and membrane biosynthesis, biological metabolism, energy metabolism, and other pathways. Then the candidate genes were screened by STRING online database and Cystoscape software, and six key genes were obtained, namely, ST8SIA5, ODC1, LAPTM5, NPC2, SNAP29, and FCGR3B.

*α*-2, 8-sialyltransferase 5 (ST8SIA5) mediates the transfer of sialic acid through the *α*-2pyrine 8-chain. Sialic acids have been reported to be involved in a variety of biological processes, including cell-cell adhesion, immune defense, tumor cell metastasis, and inflammation [36]. These biological processes also participate in the occurrence and development of atrial fibrosis and atrial remodeling. According to some researches, ST8SIA4 can promote the proliferation, migration, and invasion of thyroid cancer cells by activating PI3K-AKT-mTOR signaling pathway [37]. Sialyltransferase can also catalyze the transfer of sialic acid to proteins and lipids and participates in the synthesis of oligosaccharide core structures [38]. Natural sialylation is very important for the function of therapeutic proteins because it affects the physical, chemical, and immunogenicity of glycoproteins, and more importantly, it affects the properties of extracellular matrix to lead to atrial fibrosis.

Lysosomal-associated protein transmembrane 5 (LAPTM5) [39], Niemann-Pick C2 protein (NPC2) [40], and synaptosomal-associated protein 29 (SNAP29) [41] have the most characteristics of autophagy. Autophagy is a dynamic process regulated by multiple genes and molecular signals. The formation of autophagosomes, the transport of autophagy substrates to lysosomes and the degradation of autophagosomes in lysosomes are called autophagy energy fluxes. Autophagy is an important metabolic pathway to maintain homeostasis in eukaryotic cells under starvation, inflammation, and hypoxia/reoxygenation injury. Autolytic corpuscles mainly eliminate aging organelles and misfolded proteins and provide energy for cells. Autophagy is maintained at a low level in normal myocardium [42]. However, myocardial energy metabolism is disturbed, including myocardial injury caused by atrial fibrillation, and autophagy may be overactivated or inhibited [43]. Low-level autophagy is an important method to maintain cardiomyocyte homeostasis, that is, any form of myocardial injury will lead to cardiomyocyte autophagy. And excessive activation or inhibition of autophagy will lead to myocardial injury. Therefore, LAPTM5, NPC2, and SNAP29 may lead to atrial remodeling through myocardial injury caused by autophagy.

In addition, some studies have found that LAPTMs can act on the fibroblasts of type IV mucoliposomal disease and cause the disease. The analysis of fibroblasts of type IV mucin liposome disease shows that there are a large number of vacuolar structures, including a large number of mucopolysaccharides and lipids. Changes in the composition of extracellular matrix can lead to fibrosis [44]. LAPTMs may also cause changes in myocardial extracellular matrix components and lead to atrial fibrosis. In addition, the study also found that the structure and function of LAPTMs family is similar to mucin 1, which is known as transient receptor potential superfamily. This is an inward rectifier channel, and the change of its activity will affect the plasma levels of calcium, sodium, and magnesium ions [45]. It has also been found that injection of overexpressed NPC2 into mice through adeno-associated virus serotype 9 can lead to the accumulation of fibroblasts, and it has also been found that NPC can affect Purkinje cells, and which are also involved in cardiac electrophysiological activities [46]. More importantly, the main function of NPC is to affect the transport of cholesterol and low density lipoprotein, so it plays an important role in cardiovascular disease [47].

Ornithine decarboxylase 1 (ODC1) is mainly involved in the metabolism of polyamines, which regulates cell proliferation and differentiation. Some studies have shown that ODC1 can participate in inflammatory response after macrophage stimulation [48]. This is consistent with the presence of a large number of inflammatory cells around the myocardium in patients with atrial fibrillation, which indicates that ODC1 may participate in atrial fibrosis through inflammatory reaction and lead to atrial fibrillation. FCGR3B is a gene encoding FC-*γ* receptor 3B, which is mainly involved in immune regulation, inflammation, and cytotoxicity. Some studies have found that FCGR3B can lead to pulmonary fibrosis through proinflammatory and fibrogenic processes, including tumor necrosis factor-*α*, transforming growth factor-*β*, MCP-1, and IL-8 [49]. Although there are no reports about the direct relationship between FCGR3B and atrial fibrillation, the mechanism of atrial fibrosis in atrial fibrillation mentioned above is consistent with the mechanism of pulmonary fibrosis caused by FCGR3B, so FCGR3B may be a potential biomarker for the maintenance of atrial fibrillation.

In this study, not only six key genes were screened but also the regulatory factors of key genes, TFs and microRNAs, were predicted. Widely found across species, microRNA (miRNA, miR) is a highly conserved noncoding RNA that is composed of 19~26 nucleotides [50]. Because miRNA can regulate the expression of nearly 1/3 of all protein coding genes in the human genome, it has become an important area of research in a variety of cardiovascular disease, including atrial fibrillation. The gene that contains the miRNA coding sequence is called the miRNA host gene (HG). Because miRNA originates from posttranscriptional splicing of its host gene and may affect its host gene's expression due to their innate complementary sequences, there is crosstalk between a miRNA and its host gene. Therefore, the studies of miRNA and its host gene may provide a theoretical basis for revealing the mechanism of AF [51]. Some studies have found that microRNA-1 k affects the level of IK-1 by regulating Kir-2. It is well known that the upregulation of IK-1, which is responsible for the inward-rectifier potassium channel, is one of the important mechanisms for maintaining atrial fibrillation [52]. Meanwhile, the expression levels of miR-21 and miR-29 also confirmed that they were involved in the maintenance of atrial fibrillation [53, 54]. To this end, we also use an online database to predict the microRNAs of the six hub genes in Table 4. Finally, our results also found that the main regulatory factors of EIF5A2, HIF1A, ZIC2, ELF1, and STAT2, which target key genes, were significantly associated with valvular atrial fibrillation.

In summary, through bioinformatics, we found that autophagy, energy metabolism, ion channel, oxidative stress, and inflammatory reaction may play important roles in the occurrence and maintenance of atrial fibrillation through a variety of physiological or pathophysiological processes. Based on network regulation, we also revealed potential therapeutic targets for VAF. We also obtained six hub gene markers involved in the occurrence and maintenance of atrial fibrillation, which were statistically significant, including ST8SIA5, ODC1, LAPTM5, NPC2, SNAP29, and FCGR3B. Most of these genes are related to lysosomal autophagy, which provides new insights into the molecular mechanism of occurrence and development of atrial fibrillation. Finally, our results also confirmed that the main regulatory factors, EIF5A2, HIF1A, ZIC2, ELF1, and STAT2, are significantly associated with the occurrence and maintenance of atrial fibrillation through targeting candidate genes. Of course, microRNAs corresponding to candidate genes are also predicted, which may also be potential markers of valvular atrial fibrillation.

## 5. Limitation

There are still some limitations in our research. First of all, our results are based on microarray analysis of gene expression values, and then protein network construction is carried out. However, this is not directly equivalent to protein expression, so the biomarker in this study should be gene, not protein. What's more, it should be verified in vitro, in vivo, and clinical trials, rather than just limited to network prediction.

## 6. Conclusions

The results found that these hub genes, NPC2, ODC1, SNAP29, LAPTM5, ST8SIA5, and FCGR3B, play a key role in the development and maintenance of VAF, and their enrichment pathways and TFs elucidate the involved molecular mechanisms and assist in the validation of drug targets.

## Figures and Tables

**Figure 1:** Differential expression genes (DEGs). (a) Volcano map, *Y*-axis represents *P* value, *X*-axis represents multiple changes, each point represents a gene, and red and black represent up-down genes; (b) heat map of differentially expressed genes; and (c) sample name map.

**Figure 2:** Construction of weighted gene coexpression network (WGCN) and gene module analysis for patients with atrial fibrillation and sinus rhythm accompanied by severe mitral regurgitation: (a) gene coexpression module diagram based on dynamic branching method; (b) value of module dependency of dynamic branch cutting method (when power value is 12, independent area rises to 0.8); (c) the relationship between gene coexpression module and clinical traits. Red represents positive correlation and green represents negative correlation. (d) Connectivity of characteristic genes, with the decrease of red, the positive correlation is weaker. (e) Principal component analysis (PCA) of the two key modules, MElightcyan and MEturquoise. MEturquoise first principal component: 67.2%, second principal component: 4.1%; MElightcyan first principal component: 59.4%, second principal component: 6.4%; genetic significance (GS), module membership (MM), and activity analysis of key modules related to atrial fibrillation in (f) and (g).

**Figure 3:** Key module DEGs gene ontology (GO) analysis. (a, b) GO analysis of DAVID database MElightcyan and MEturquoise module gene, dot size represents the number of genes contained, dot color represents *Q* value.

**Figure 4:** The KEGG analysis of the key module DEGs: (a, b) the enrichment analysis in the Metascape database, the circle size represents the size of the Log*P* value, and the color represents the enrichment fraction.

**Figure 5:** DEGs protein-protein interaction network map and key gene screening maps. (a) and (h) represent the PPI of DEGs in which the MElightcyan and MEturquoise modules related to pathways of atrial remodeling and fibrosis, such as energy metabolism, biosynthesis, ion channels, cytoskeleton, and vesicle secretion. (b)–(g) represent modules 1~5 obtained by MCODE plugin analysis of the DEGs protein interaction network of the MElightcyan, in which red represents the central node, namely, the key gene of the corresponding module.

**Figure 6:** Box plot diagram of hub gene expression in atrial fibrillation and sinus patients and left and right atrial tissues.

**Figure 7:** The violin plot diagram of hub gene expression level between atrial fibrillation and sinus rhythm patients: (a)–(f) represent the differences in the expression levels of the six hub genes, ST8SIA5 (*P* = 6.9*e* − 16), ODC1 (*P* = 7.9*e* − 08), LAPTM5 (*P* = 7.1*e* − 07), NPC2 (*P* = 2.2*e* − 06), SNAP29 (*P* = 2.7*e* − 10), and FCGR3B (*P* = 4.7*e* − 11), in patients with atrial fibrillation and sinus diseases, with *P* values less than 0.05, which are of significant statistical significance.

**Figure 8:** Prediction of transcription factors of hub gene: green indicates the top five transcription factors with the highest standard enrichment score, red indicates the hub gene, and arrows indicate the degree of association between TFs and hub gene.

**Table 1:** Top 5 up- and downregulated genes of chip GSE115574.

Gene ID	logFC	AveExpr	*t*	*P* Value	Adj.*P*.Val	B
RGS6	0.516701	4.290465	9.958301	2.64*E* − 14	2.27*E* − 12	22.2945
OTOGL	1.275203	5.172998	7.768166	1.26*E* − 10	2.37*E* − 09	13.94223
KIAA0753	0.551188	5.603697	7.504565	3.53*E* − 10	5.69*E* − 09	12.92274
PCDHGA10	0.936869	4.489173	7.259196	9.26*E* − 10	1.28*E* − 08	11.97422
LOC100506813	0.653479	5.248975	6.776567	6.13*E* − 09	6.37*E* − 08	10.11424
FCGR3B	-1.26104	3.645921	-24.147	1.66*E* − 32	3.41*E* − 28	62.87675
CTNS	-0.61385	4.013762	-17.8101	1.44*E* − 25	1.11*E* − 21	47.67246
SLC35E1	-0.60841	5.726716	-17.7658	1.63*E* − 25	1.11*E* − 21	47.55132
TIFAB	-0.74335	3.823311	-17.3504	5.35*E* − 25	2.74*E* − 21	46.40393
ARHGAP22	-0.61343	3.371978	-16.8357	2.39*E* − 24	9.80*E* − 21	44.95354

**Table 2:** The KEGG network pathway terms of key modules.

Modules	Description	Gene	Log*P*
MElightcyan	mTOR signaling pathway	ATP6V1B2, CHUK, PRKAA2, MAP2K1, RPS6KA2, RPS6KA3, etc.	-5.10575
	Fc epsilon RI signaling pathway	GFPT1, HEXB, HK1, etc.	-4.82544
	Autophagy-animal	PRKAA2, SNAP29, SH3GLB1, etc.	-3.22867
	Proteasome	PSMC4, PSMD7, PSMD8,etc.	-2.80551
	Lysosome	ATP6AP1, HEXB, LAPTM5, etc.	-2.58718
	Natural killer cell-mediated cytotoxicity	ARAF, FCER1G, IFNGR2, ITGB2, etc.	-2.41921
	Insulin signaling pathway	ARAF, HK1, PRKAA2, etc.	-2.34109
	Glycosaminoglycan biosynthesis, heparan sulfate backbone	EXT1, EXT2	-2.28058
	SNARE interactions in vesicular transport	STX4, SNAP29, YKT6	-2.19845
MEturquoise	Natural killer cell-mediated cytotoxicity	FCGR3B, ITGAL, HCST	-2.70881
	Glycosaminoglycan biosynthesis, heparan sulfate backbone	EXTL3	-1.73339
	O-glycan biosynthesis, mucin type core	GALNT10	-1.30872
	Lysosome	CTNS, CTSV	-1.65612
	*Staphylococcus aureus* infection	C2, FCGR3B, ITGAL	-3.80614

**Table 3:** TFs of top five enrichment fractions.

TF	NES	Target	Motif
EIF5A2	12.134	4	2
HIF1A	8.032	6	91
ZIC2	7.489	6	4
ELF1	7.474	2	7
STAT2	6.947	5	6

**Table 4:** Functional analysis and microRNA prediction of hub genes.

Hub gene	MicroRNAs	Functional		*P* value
ST8SIA5	miR-218-5p miR-203a-3p.1 miR-218-5p miR-4295 miR-3666 miR-301a-3p	KEGG	Glycosphingolipid biosynthesis, ganglio series, LacCer = > GT3	0.019
		GO	Golgi apparatus Golgi membrane	0.0004 0.0001
ODC1	miR-188-5p miR-6866-3p miR-133a-3p miR-3184-5p	KEGG	Polyamine biosynthesis, arginine = > ornithine = > putrescine	0.014
		GO	Cytoplasm Cytosol	2.0 E-06 0.0001
LAPTM5	Hsa-miR-330-3p Hsa-miR-6766-3p Hsa-miR-219a-5p Hsa-miR-4782-3p	KEGG	Lysosome mTOR signaling pathway	0.019 0.05
		GO	Membrane Proteasome accessory complex	0.00007 0.006
NPC2	Hsa-miR-23c Hsa-miR-23a-3p Hsa-miR-130a-5p Hsa-miR-23b-3p	KEGG	Lysosome Amino sugar and nucleotide sugar metabolism	0.0258 0.04
		GO	Endoplasmic reticulum	0.049
			Extracellular exosome	0.0107
SNAP29	miR-338-3p miR-124-3p Hsa-miR-222-3p Hsa-miR-221-3p	KEGG	SNARE interactions in vesicular transport Autophagy-animal	0.024 0.03
		GO	Golgi membrane Autophagosome membrane	4.69E-4 0.0045
FCGR3B	Hsa-miR-6893-3p Hsa-miR-370-3p	KEGG	Natural killer cell mediated cytotoxicity Staphylococcus aureus infection	0.027 0.038
